# A Retrospective Study of Diaphragmatic Breathing Training Combined with Discharge Care Bundles in Patients with Chronic Obstructive Pulmonary Disease

This article has been retracted.

**DOI:** 10.1155/2022/9649986

**Published:** 2022-09-14

**Authors:** Shuhui Yu, Chen Lu, Lingling Qin

**Affiliations:** Respiratory Department, Huzhou Central Hospital & Affiliated Central Hospital, HuZhou University, Huzhou, China

## Abstract

**Objective:**

Both physical exercise and discharge care bundles can improve patient outcomes and reduce hospitalization rates among subjects with chronic obstructive pulmonary disease (COPD). The retrospective analysis aims to determine the advantages of care bundles combined with diaphragmatic breathing training (DBT) in COPD patients after discharge.

**Methods:**

Of the 110 COPD patients, 55 patients received DBT alone (DBT group) and 55 participants received the combined intervention (care bundle + DBT group). Three months after discharge, we assessed the outcomes of patients using Bristol COPD Knowledge Questionnaire (BCKQ), Hospital Anxiety and Depression Scale (HADS), COPD Assessment Test (CAT), and St. George's Respiratory Questionnaire (SGRQ). Meanwhile, COPD-related hospital readmissions were also recorded.

**Results:**

The BCKQ score for assessing the disease knowledge level was increased in patients at 3 months after the combined interventions as compared to the baseline values, which was higher in the care bundle + DBT group than the DBT group at 3 months. Moreover, improvements in negative emotion and clinical symptoms from baseline to 3-month follow-up were seen in both the two groups. Besides, the care bundle + DBT group showed the mitigation of depression and anxiety and the alleviation of clinical symptoms in comparison with the DBT group at 3 months. Participants who received combined interventions had lower SGRQ scores than those who received DBT alone. The time to first COPD-related readmission was shorter for patients in the care bundle + DBT group compared with the DBT group.

**Conclusions:**

DBT combined with discharge care bundles for COPD patients resulted in improvements in disease-specific knowledge, negative emotions, and clinical symptoms with better HRQOL and lower readmission rate.

## 1. Introduction

Chronic obstructive pulmonary disease (COPD) is a chronic progressive respiratory disease that leads to irreversible airway obstruction, with a high global prevalence of about 20.9%, and it is responsible for the leading cause of death worldwide [1]. In 2016, COPD was the fifth leading cause of death in China with the prevalence ranging from 2% to 21% [2]. Patients with COPD often show a series of symptoms such as coughing, dyspnea, wheezing, and chest tightness [3]. Furthermore, compared with the general population, COPD patients are frequently attacked by cardiovascular and metabolic diseases [4], lung cancer [5], anxiety, and depression [6], which significantly diminish the quality of life and increase health resource utilization [7, 8]. Furthermore, approximately one-third of COPD patients were reported to be readmitted within 90 days of discharge, resulting in 13.9% of death [9]. The good thing is that the management of COPD has improved, including early detection and treatment and primary care practice.

Currently, as a kind of low-intensity aerobic exercise, diaphragmatic breathing training (DBT) with special breathing techniques is a commonly used intervention in pulmonary rehabilitation [10]. DBT contributes to alleviate dyspnea, improve pulmonary function and enhances health-related quality of life in patients with COPD by increasing the strength and endurance of respiratory muscles along with diaphragmatic excursion, reducing accessory muscle use, and guiding the correct breathing patterns [10–12]. As reported in some studies, DBT has been extremely beneficial for increasing tidal volume, reducing respiratory rate, and improving breathing patterns [13, 14]. Moreover, DBT intervention as a home-based pulmonary rehabilitation was reported to be feasible in COPD patients, with high retention and adherence [15, 16].

Care bundles, consisting of a series of structured evidence-based interventions, aimed to improve patient recovery and outcomes, and have been applied to various diseases that include bloodstream infections [17], postpartum hemorrhage [18], and ventilator-associated pneumonia in pediatrics [19]. As for COPD patients, care bundles were reported to be used as an effective approach for improving the quality of life and reducing mortality after discharge [20, 21]. However, evidence to explore the efficacy of DBT combined with care bundles in COPD patients remains to be elucidated.

The retrospective study enrolled 110 patients diagnosed with COPD and assigned them into two groups, receiving DBT alone and DBT combined with care bundles, respectively. The aim of our study is to assess the superiority of the combination treatment in terms of disease-related knowledge mastery, clinical symptoms, and readmission rates in COPD patients after discharge.

## 2. Methods

### 2.1. Study Population

Participants (*n* = 110) with a primary diagnosis of moderate to severe COPD by a pulmonologist or spirometry were recruited in this retrospective study according to the Global Initiative for Chronic Obstructive Lung Disease (GOLD) criteria [22] (Table 1), who were able to read, write, and speak. Moreover, all patients had stable respiratory conditions without changes in medication or symptoms for at least 4 weeks, and they were given regular treatment with inhaled bronchodilators and steroids. The exclusion criteria were as follows:: (1) diagnosis of cancer; (2) presently attending a pulmonary rehabilitation course or other similar COPD education course; (3) diagnosis of developed serious cardiopulmonary, neuromuscular disease, or dementia; (4) previous engagement in any exercise training program in the prior 2 years; and (5) drug abuse or alcohol abuse. Of these 110 COPD patients, 55 patients received DBT alone (DBT group) and 55 participants received the combined intervention (care bundle + DBT group). All patients completed the baseline and 3-month follow-up assessments. The flow diagram of participants in this retrospective study is illustrated in Figure 1.

### 2.2. DBT Program

At discharge, all patients in the care bundle + DBT group and the DBT group were instructed on how to complete a DBT program according to previous studies [12, 23]. The DBT program consisted of three 45-minute weekly sessions for 3 months. The patients performed a total of 150 breathing exercises in each session in the five positions (supine, right lateral decubitus, left lateral decubitus, sitting, and standing) with 3 series of 10 repetitions in each position. These exercises were taught to patients in detailed face-to-face sessions held on three successive days as to how to carry out the DBR intervention at home. The patients would receive a telephone call to remind them of doing the breathing exercises.

### 2.3. COPD Discharge Care Bundles

Except for the DBT exercises, the patients in the care bundle + DBT group also received the discharge care bundles for 3 months of follow-up based on the previous studies [24, 25], including adequate assessment of the patient's understanding on the use of medications and effective inhaler technique, educational programme on disease management, referral for pulmonary rehabilitation, arrange outpatient follow-up in the respiratory clinic, referral to a smoking-cessation programme, and 3- month telephone calls from respiratory nurses.

### 2.4. Assessment of the Knowledge Level in COPD Patients

The disease-specific knowledge level of patients with COPD was assessed using the Bristol COPD Knowledge Questionnaire (BCKQ) with a total score ranging from 0 to 65 (higher scores indicate greater knowledge of COPD) [26]. The BCKQ was composed of 13 domains, and each domain with five statements giving a total of 65 questions for which there is a response option of “true,” “false,” and “do not know”. Correct and wrong responses are scored as “1” and “0”, respectively.

### 2.5. Assessment of the Negative Emotion and Clinical Symptoms in COPD Patients

The Hospital Anxiety and Depression Scale (HADS) was used to determine the negative emotion (anxiety and depression) in patients with total scores ranging from 0 to 21. The clinical symptoms in patients were determined by the COPD Assessment Test (CAT) [27]. It comprises 8 questions, each presented as a semantic 6-point (0–5) differential scale, providing a total score out of 40.

### 2.6. Assessment of Health-Related Quality of Life (HRQOL) in COPD Patients

The St. George's Respiratory Questionnaire (SGRQ) was used to evaluate COPD-specific HRQOL [28], which has 50 topics with four scores, including total, symptoms, activity, and impact. Each score ranged from 0 to 100. The higher SGRQ score indicated the worse possible HRQOL.

### 2.7. Readmission Rate

Readmission data included inpatient, emergency department, and outpatient (classified as a short stay or 24-hour observation and not admitted as inpatients); hospital admissions [29] were obtained through electronic health records even if the patient did not complete the study calls. The time to first COPD-related readmission was recorded to determine the impact of the intervention on patient outcomes.

### 2.8. Statistical Analysis

Sample size was calculated based on the SGRQ scores in COPD patients after the intervention (effect size = 0.492; *α* error = 0.05, power = 0.8). To account for possible 5% losses to follow-up, 55 patients with COPD in each group had to be recruited. A *P* < 0.05 was considered to indicate a statistical significance in all analyses, which were performed in GraphPad Prism. In order to investigate the distribution of data, we employed the Shapiro–Wilk test, and all data were expressed as mean ± SD for variables with parametric distributions in our study. The comparison of measurement data and counting data (*n*) was done using the student's *t* test for unpaired or paired samples and the *χ*^2^ test, respectively.

## 3. Result

### 3.1. Baseline and Clinical Characteristics of COPD Patients

The basic information of the patients in the care bundle + DBT group (*n* = 55) and DBT group (*n* = 55) are listed in Table 2. There were no statistically significant differences between both the groups regarding the age (*P*=0.274), sex (*P*=0.525), BMI (*P*=0.725), COPD duration (*P*=0.475), smoking status (*P*=0.658), COPD severity (*P*=0.558), marital status (*P*=0.463), employment status (*P*=1.000), educational level (*P*=0.109), FEV1 (%) (*P*=0.261), FEV1/FVC (%) (*P*=0.694), PaO_2_ (*P*=0.138), PaCO_2_ (*P*=0.667), and 6MWD (*P*=0.177).

### 3.2. Comparison of the Disease Knowledge Level between the Two Groups

Figure 2(a) shows no obvious difference in the overall BCKQ scores at baseline between the care bundle + DBT group and the DBT group (22.8 ± 13.24 vs. 24.78 ± 11.91, *t* = 0.825, *P*=0.411), which was increased significantly at 3 months after the combined interventions (34.65 ± 13.86 vs. 22.8 ± 13.24, *P* < 0.05). However, for the disease-specific knowledge level, no improvement was found in the DBT group from baseline to 3-month follow-up (25.71 ± 11.79 vs. 24.78 ± 11.91, *P* > 0.05). As compared with the DBT group, the patients in the care bundle + DBT group had a higher total score of BCKQ at 3 months after the interventions (34.65 ± 13.86 vs. 25.71 ± 11.79, *P* < 0.05).

### 3.3. Comparison of the Negative Emotion between the Two Groups

As demonstrated by Figures 2(b) and 2(c), the improvements in negative emotions from baseline to 3-month follow-up were seen in both the care bundle + DBT group and DBT group with reduced HADS score (both *P* < 0.05). Besides, the care bundle + DBT group showed statistically significant alleviation of depression and anxiety in comparison with the DBT group at 3 months (both *P* < 0.05). At baseline, participants in both the study groups revealed no significant differences regarding the HADS score (both *P* > 0.05).

### 3.4. Comparison of the Clinical Symptoms and HRQOL between the Two Groups

Although the difference in clinical symptoms as assessed by CAT scores between the two groups was not statistically significant at baseline (DBT group: 16.64 ± 5.76; care bundle + DBT group: 15.67 ± 8.06, *P* > 0.05), the patients after the intervention had lower CAT scores than the baseline values in both the DBT group and care bundle + DBT group. Moreover, the care bundle + DBT group (10.95 ± 6.31) experienced an obvious reduction compared with the DBT group (13.45 ± 5.69) at 3 months (*P* < 0.05, Table 3). Furthermore, the care bundle + DBT group had a slightly higher proportion of people who experienced clinically alleviated clinical symptoms than the DBT group without a statistical difference (*P* > 0.05). In addition, differences in SGRQ scores between the care bundle + DBT group (54.22 ± 16.62) and DBT group (54.40 ± 16.64) were small and statistically not significant at baseline (*P* > 0.05), but participants in the care bundle + DBT group (3652 ± 17.61) had better HRQOL (lower SGRQ scores) than those in the DBT group (45.00 ± 16.88) at 3 months (*P* < 0.05, Table 3).

### 3.5. Comparison of the Readmission Rates between the Two Groups

We found that 15 (27.27%) of 55 patients in the DBT group had at least one readmission during the course of the study compared with 6 (10.91%) of 55 persons in the care bundle + DBT group. There was an increased total number of COPD-related readmissions in the DBT group than in the care bundle + DBT group (30 cases vs. 12 cases). Kaplan–Meier analysis of the time to first COPD-related hospital readmission is presented in Figure 3. Overall, the time to first COPD-related readmission was longer for patients in the care bundle + DBT group compared with the DBT group (*χ*^2^ = 4.810, *P*=0.028), with more events occurring in the DBT group after the program completion.

## 4. Discussion

COPD is the third leading cause of death worldwide, which seriously affects human health and causes a heavy social and economic burden [30]. Breathing exercises and care bundles are widely used in the treatment of COPD, aiming to improve the physical and psychological status of COPD patients [20, 31]. As part of the pulmonary rehabilitation method (comprehensive intervention program), breathing exercises are a simple but highly targeted training that can be completed at home independently by patients with COPD, resulting in strengthening the respiratory muscle and ultimately improving long-term management of dyspnea [32, 33]. DBT is a common physiotherapy technique used to relieve dyspnea, improve pulmonary function, and enhance the psychological condition of COPD patients [34, 35]. Significant variations in readmission outcomes and provision of COPD care have been noted. Furthermore, the care bundle was associated with significant improvements in pulmonary rehabilitation, smoking cessation, and relevant knowledge of inhalers [21]. In our retrospective study, we included a total of 110 participants with a primary diagnosis of moderate to severe COPD. Among them, 55 patients were treated with DBT alone and the remaining 55 patients received DBT combined with the discharge care bundle.

In recent years, professionals have emphasized the importance of patient self-management and increased patients' want to better understand their condition. Therefore, it is particularly important to carry out medical education for patients and their families. Due to the variations in the form and content of medical education, there are differences in the results of education for COPD patients [26, 36, 37]. The BCKQ is a kind of questionnaire used to assess the knowledge of individual patients. “Incorrect” or “do not know” options indicate that patients have insufficient knowledge where specific education is needed [38]. In our study, after a 3-month intervention, we found that the overall BCKQ score of the care bundle + DBT group was significantly increased compared to the baseline data. White et al. implied that the average BCKQ scores of COPD patients was 54.7% before education but the score was increased to 73%, which was maintained for six months in most patients, following an eight-week education programme [26].

COPD patients are more likely to suffer from psychological diseases including depression and anxiety, which might induce poor treatment compliance [6]. Hence, we evaluated the psychological condition of the two groups through the HADS score. The HADS has been developed as a simple measurement of clinical symptoms of depression, anxiety, and fear in patients with mental diseases [39]. HADS has been widely used in lung-related diseases including lung cancer [40], thromboembolism [41], and pneumonia [42]. Compared with the baseline, the care bundle + DBT group and DBT group both the groups revealed reduced HADS scores, indicating alleviation in negative emotion after interventions. In addition, a significantly lower HADS score was found in the care bundle + DBT group than that of the DBT group at 3 months.

The present study also assessed clinical symptoms via CAT scores and COPD-specific HRQOL by the SGRQ score. The findings demonstrated that both the two groups had reduced CAT scores after the intervention, and this trend was more obvious in the care bundle + DBT group. People with specific diseases are related to an increased risk of death, and these diseases may lead to dysfunction and symptoms, affecting personal activities of daily living. HRQOL terms are often used specifically to assess the health status of individuals with diseases that impair daily functions or cause symptoms [43]. Our study observed that the patients with care bundle + DBT intervention had lower SGRQ scores compared to the DBT group, suggesting care bundle + DBT intervention improved HRQOL.

It has been proposed that the care bundle is an effective method to prevent COPD readmission after hospitalization, reducing the 30-day all-cause readmission rate from 22.7% to 14.7% [28]. As reported by Laverty et al. discharge care bundle has an advantage in the reduction in the readmission rate of COPD [9]. Fewer patients in the care bundle + DBT group were readmitted to the hospital compared to the DBT group. Furthermore, Kaplan–Meier analysis indicated that the patients in the care bundle + DBT group showed a longer time of first COPD-related readmission than that in the DBT group. Of note, some limitations were presented in our study, for instance, 3-month follow-up may not be enough to evaluate the long-term efficacy of the combined intervention. Besides, we need a large number of subjects to verify our findings. Furthermore, fatigue is one of the most disabling symptoms of COPD [44], and COPD was reported to result in poor cardiopulmonary endurance [45], indicating fatigue level and cardiopulmonary should be taken into consideration in future analysis. The explanations of abbreviations in this study have been listed in Supplementary Table 1.

To sum up everything, DBT combined with the discharge care bundle appeared to be associated with improvement in disease-specific knowledge levels and a reduction in readmission rate. Combined intervention is superior to the DBT intervention alone in terms of assessment of depression and anxiety, clinical symptoms, and HRQOL.

## Figures and Tables

**Figure 1:** The flow diagram of participants in this retrospective study.

**Figure 2:** Comparison of the disease knowledge level and negative emotions between the two groups. (a) The disease-specific knowledge level of patients with COPD was assessed using the Bristol COPD Knowledge Questionnaire (BCKQ); (b)-(c): Hospital Anxiety and Depression Scale (HADS) was used to determine the negative emotion (anxiety and depression) in COPD patients.

**Figure 3:** Kaplan–Meier analysis of the time to first COPD-related hospital readmission between the two groups.

**Table 1:** Global initiative for chronic obstructive lung disease (GOLD) of severe to moderate COPD.

Stage	Characteristics
Moderate	FEV1/FVC < 70% 50% ≤ FEV1 < 80% With or without chronic symptoms (cough and sputum production)

Severe	FEV1/FVC < 70% 30% ≤ FEV1 < 50% With or without chronic symptoms (cough and sputum production)

**Table 2:** The basic information of COPD patients in the care bundle + DBT (*n* = 55) and the DBT group (*n* = 55).

Parameter	DBT group	Care bundle + DBT group	*P*
*Age (years)*			
>60	49	45	
≤60	6	10	0.274

*Sex*			
Male	41	38	
Female	14	17	0.525

BMI (kg/cm^2^)	21.09 ± 1.74	20.96 ± 1.87	0.725

COPD duration (years)	3.13 ± 1.29	2.95 ± 1.37	0.475

*Smoking status*			
Current	30	28	
Former	11	15	
Never	14	12	0.658

*COPD severity*			
Moderate	35	32	
Severe	20	23	0.558

*Marital status*			
Single	5	3	
Married	50	52	0.463

*Employment status*			
Employed	3	3	
Retired	52	52	1.000

*Educational level*			
≤9 years	32	40	
>9 years	23	15	0.109

FEV1 (%)	54.85 ± 13.59	52.00 ± 12.91	0.261

*FEV1/FVC (%)*	56.27 ± 6.95	55.76 ± 6.59	0.694
PaO_2_	63.25 ± 7.20	61.07 ± 8.08	0.138
PaCO_2_	37.44 ± 5.36	37.89 ± 5.68	0.667
6MWD	381.73 ± 118.95	414.58 ± 134.17	0.177

**Table 3:** Comparison of the clinical symptoms by CAT scores and HRQOL by SGRQ scores between the two groups.

Groups	*CAT scores*			*SGRQ scores*		
	Before	After	*P*	Before	After	*P*
DBT group	16.64 ± 5.76	13.45 ± 5.69	<0.001	54.40 ± 16.64	45.00 ± 16.88	<0.001
Care bundle + DBT group	15.67 ± 8.06	10.95 ± 6.31	0.003	54.22 ± 16.62	36.52 ± 17.61	<0.001
*P*	0.866	0.027		0.954	0.024	

## Data Availability

The data used to support the findings of this study are included within the article.

## Supplementary Materials

Supplementary Materials The explanations of abbreviations in this study have been listed in Supplementary Table 1.
